# Collateral Status and Clinical Outcomes after Mechanical Thrombectomy in Patients with Anterior Circulation Occlusion

**DOI:** 10.1155/2022/7796700

**Published:** 2022-01-25

**Authors:** Yuzhu Xu, Songtao Guo, Hao Jiang, Hui Han, Jian Sun, Xi Wu

**Affiliations:** Department of Neurosurgery, Inner Mongolia Xing'an Meng People's Hospital, Xing'an 137400, Inner Mongolia, China

## Abstract

**Background:**

Successful mechanical thrombectomy (MT) requires reliable, noninvasive selection criteria. We aimed to investigate the association of collateral status and clinical outcomes after MT in patients with ischemic stroke due to anterior circulation occlusion.

**Methods:**

109 patients with poor collaterals and 110 aged, sex-matched patients with good collaterals were enrolled in the study. Collateral circulation was estimated by the CT angiography with a 0–3 scale. The collateral status was categorized as poor collaterals (scores 0–1) and good collaterals (scores 2-3). The reperfusion was assessed by the modified Treatment in Cerebral Infarction scale (mTICI, score 0/1/2a/2b/3). The clinical outcomes included the scores on the modified Rankin scale (mRS, ranging from 0 to 6) and death 90 days after mechanical thrombectomy.

**Results:**

Patients with greater scores of collateral status were more likely to achieve successful reperfusion (mTICI 2b/3). Patients with good collaterals were significantly associated with a higher chance of achieving mRS of 0–1 at 90 days (adjusted ORs: 4.55; 95% CI: 3.17–7.24; and *P* < 0.001) and a lower risk of death at 90 days (adjusted ORs: 0.87; 95% CI: 4.0%–28.0%; and *P* = 0.012) compared to patients with poor collaterals. In subgroup analyses, patients with statin use seem to benefit more from the effect of collateral status on good mRS (≤2).

**Conclusion:**

Among patients with acute ischemic stroke caused by anterior circulation occlusion, better collateral status is associated with higher scores on mRS and lower mortality after mechanical thrombectomy. Statin use might have an interaction with the effect of collateral status.

## 1. Introduction

Over the past decades, the stroke burden has increased in China, and ischemic stroke accounted for 69.6% of incident strokes and 77.8% of prevalent strokes in 2013 [1]. Stroke is one of the leading causes of death [2], and the mortality rates at 3, 6, and 12 months after stroke are 11.3%, 14.4%, and 17.8% in women and 7.6%, 9.7%, and 12.3% in men, respectively [3]. Besides, patients after ischemic stroke often have impaired quality of life and functional capacity [4]. Mechanical thrombectomy (MT) has been consistently demonstrated to be an effective treatment for patients after ischemic stroke of anterior circulation occlusion in prospective randomized trials [5–7]. The data from another large-scale trial extended the time window after stroke from 6 to 8 hours [8]. In addition, patients after anterior circulation occlusion could also benefit from MT within 6–16 hours [9] and 6–24 hours [10] after strict imaging screening, well beyond the time window of 6 hours. The abovementioned evidence suggests that other factors may contribute to the clinical outcome of patients after anterior circulation occlusion in MT besides the time window.

The brain's collateral circulation is defined as the arterial anastomotic pathways that are capable of providing nutrient perfusion to an impaired brain region when blood flow has become compromised by disease [11]. The Willis circle, one of the most essential components of the cerebral collateral circulation, may have substantial variability in the size and degree of completeness in normal individuals [12]. Previous studies indicated that the status of cerebral collateral circulation, whether estimated by digital subtraction angiography (DSA) [13] or CT angiography (CTA) [14, 15], is significantly associated with functional outcomes in patients treated with MT. Good collateral circulation can sustain ischemic penumbra until reperfusion occurs, preventing the growth of cerebral infarction [16]. However, previous studies on the association of collateral flow and clinical outcomes showed inconsistent results. In a study of 1412 patients with anterior circulation occlusion treated by endovascular therapy, good collateral status was associated with good functional independence and low mortality [17]. Another study also showed that better collaterals were associated with a greater likelihood of successful reperfusion (*P* = 0.019) [18]. In contrast, a previous retrospective study did not find a significant association between collateral status (odds ratio: 1.681 and 95% confidence intervals: 0.683–4.140) and successful reperfusion [19].

In this study, we aimed to determine whether mechanical thrombectomy would be associated with successful reperfusion, functional outcomes, and death in patients who had large-vessel occlusion in the anterior circulation. We further investigated the factors which modified the effect of mechanical thrombectomy on clinical outcomes.

## 2. Methods

### 2.1. Study Population

This study was a prospective, observational study, and we recruited patients aged ≥18 years from January 2015 to December 2018. The inclusion criteria for patients were as follows: patients who had an acute ischemic stroke due to large-vessel occlusion in the anterior circulation, as confirmed by computed tomographic angiography (CTA) and a score of 1 or less on the modified Rankin scale (ranging from 0 to 6) if they had previously had a stroke. Patients with the following conditions were excluded: a disability before the ischemic stroke; and severe concomitant diseases that may affect the outcomes. Our hospital performed at least 60 mechanical thrombectomy procedures every year, and every mechanical thrombectomy in this study was performed by trained and experienced neurologists according to the guidelines from the American Heart Association/American Stroke Association [20]. Finally, 109 patients in the poor collateral group and 110 aged, sex-matched patients in the good collateral group were enrolled in the study. We continuously included patients with anterior circulation occlusion in our hospital, and then the patients were categorized into two groups based on a similar proportion of age and sex. Finally, the two groups of patients were matched by age and sex. Written informed consent was obtained from all the participants before data collection. The study protocol was approved by the medical ethics committee.

### 2.2. Clinical Data Collection and Imaging Assessment

The trained healthcare providers collected the clinical data on a standardized form in face-to-face interviews with patients and their family members. The data included age, sex, history of diseases, medication use, systolic blood pressure (SBP) and glucose at hospital arrival, time from stroke onset to intravenous alteplase, time from stroke onset to groin puncture, time from stroke onset to revascularization, and location of intracranial artery occlusion. The neurologic deficit was estimated by a score on the National Institutes of Health Stroke Scale (NIHSS, ranging from 0 to 42), with higher scores suggesting more severe deficits.

The evaluation of all CTA data was accomplished by two experienced and trained neuroradiologists, and a third reader would solve the discrepancies between the two readers. Collateral circulation was estimated by the CTA with a 0–3 scale: 0 for absent collateral circulation, 1 for collateral supply filling >0% and ≤50% of the occluded territory, 2 for collateral supply filling >50% and <100% of the occluded territory, and 3 for collateral supply filling 100% of the occluded territory [21]. The collateral status was categorized as poor collaterals (scores 0–1) and good collaterals (scores 2–3). The reperfusion after mechanical thrombectomy was assessed by the modified Treatment in Cerebral Infarction scale (mTICI, score 0/1/2a/2b/3), and the mTICI 0/1/2a was defined as unsuccessful reperfusion, the mTICI 2b/3 as successful reperfusion [22].

### 2.3. Clinical Outcomes

Experienced neurologists conducted the follow-up interviews to evaluate clinical outcomes at 90 days by face-to-face visits or telephone with the patient or family member. The clinical outcomes included the scores on the modified Rankin scale (mRS) and death 90 days after mechanical thrombectomy. The scores on the mRS ranged from 0 to 6, with 0 suggesting no symptoms at all; 1, no significant disability; 2, slight disability; 3, moderate disability; 4, moderately severe disability; 5, severe disability; and 6, death [23]. Functional independence was defined as good mRS (≤2).

### 2.4. Statistical Analysis

All the analyses were performed between two groups: poor collaterals and good collaterals. Continuous variables were presented as mean ± SD, or median (interquartile range, IQR), and compared by the Student's *t*-test or nonparametric test. Categorical variables were expressed as *n* (%), and compared by the Chi-square test. The degree of reperfusion and the distribution of scores on mRS were analyzed between the poor collateral group and the good collateral group. Odds ratios (ORs) and 95% confidence intervals (95%CIs) were used to estimate the effect of collateral status on the scores of mRS (0–1 versus 2–6; 0–2 versus 3–6; 0–3 versus 4–6; and 0–4 versus 5–6) and mortality at 90 days by logistic regression analysis, with adjustment for potential confounding factors. We further analyze the effect of collateral status on good mRS (≤2) by subgroups, including age, history of ischemic stroke, statin use, SBP and NIHSS at hospital arrival, and location of intracranial artery occlusion. A two-tailed value of *P* < 0.05 was considered statistically significant. Figures were drawn using GraphPad Prism 6.0. All the analyses were performed by SPSS Statistics 21.0 (IBM SPSS, Armonk, NY).

## 3. Results

A total of 219 patients were enrolled in the study, including 109 patients in the poor collateral group and 110 in the good collateral group. The mean ± SD age of 219 patients was 67.7 ± 8.5 years, and 53.9% (118) of them were male. The clinical characteristics of patients by collateral status are shown in Table 1. Age and sex were comparable in these two groups. Compared with the poor collateral group, patients with good collaterals were likely to have a lower prevalence of hypertension, diabetes, ischemic stroke, higher rates of statin use, and lower SBP levels and NIHSS at hospital arrival. Besides, patients with good collaterals seem to have better clinical outcomes, including higher rates of good mRS (≤2) and reduced mortality at 90 days, compared to individuals with poor collaterals. No significant differences were found in history of atrial fibrillation, antiplatelet medication use, anticoagulant drug use, glucose at hospital arrival, time from stroke onset to intravenous alteplase, time from stroke onset to groin puncture, and time from stroke onset to revascularization between the two groups (Table 1).

The degree of reperfusion stratified by collateral status is illustrated in Figure 1. Individuals with greater scores of collateral status more frequently achieved successful reperfusion (mTICI 2b/3). Among the patients with the poorest collateral status (0 score), successful reperfusion (mTICI 2b/3) was achieved in 67% of patients, whereas it was observed in 72% of patients with a collateral status of 1 score, 75% of patients with a collateral status of 2 scores, and 82% of patients with a collateral status of 3 scores (*P* < 0.001).

Figure 2 shows the scores on the modified Rankin scale (mRS) for the subjects in the two groups. Of patients with poor collaterals, 47.7% were functionally independent (mRS ≤2) at 90 days, whereas 58.1% of patients with good collaterals were functionally independent. Individuals in the poor collateral group had a higher mortality than patients in the good collateral group at 90 days (26.6% versus 20.0%). Briefly, patients with good collaterals seem to have a better functional outcome compared to patients with poor collaterals.

We found a significant modification effect of collateral status on the clinical outcomes including both mRS and mortality at 90 days, adjusted for age, history of diseases, medication use, SBP at hospital arrival, location of intracranial artery occlusion, and the NIHSS at hospital arrival (Table 2). As illustrated in Table 2, patients with good collaterals had a 355% (95% CI: 217%–624%) absolute increase in the chance of achieving mRS of 0–1 at 90 days compared to patients with poor collaterals (adjusted ORs: 4.55; 95% CI: 3.17–7.24; and *P* < 0.001). Mortality at 90 days was 26.6% in the poor collateral group and 20.0% in the good collateral group. Compared to patients with poor collaterals, the absolute decrease of risk for death was 13.0% (95% CI: 4.0%–28.0%; adjusted ORs: 0.87; and *P* = 0.012) in patients with good collaterals.

In Table 3, we further performed the subgroup analysis in the effect of collateral status on good mRS (≤2). No significant differences in the effect of collateral status were detected across the subgroups of age, SBP, and NIHSS at hospital arrival, and location of intracranial artery occlusion. Of interest, patients with a history of ischemic stroke and statin use seem to benefit more from the effect of collateral status on good mRS. However, the small sample size may reduce the power of these subgroup analyses.

## 4. Discussion

In patients with acute ischemic stroke caused by anterior circulation occlusion who were eligible for treatment with mechanical thrombectomy, better collateral status led to improved clinical outcomes, including the scores on the mRS and mortality. Besides, patients with greater scores of collateral status were more likely to achieve successful reperfusion (mTICI 2b/3). In subgroup analyses, we found that history of ischemic stroke and statin use may have contributed to the effect of collateral status on good mRS.

Previous studies have demonstrated the importance of collateral status as a predictive factor on clinical outcomes in patients with ischemic stroke. In a post hoc analysis of the Interventional Management of Stroke (IMS) III trial, maximal benefit was seen in patients with intermediate collateral status and none in patients with poor collateral status assessed by the CTA [24]. In a meta-analysis of 34 studies enrolling 5768 patients, good collateral status was independently associated with successful reperfusion and functional independence (RR: 1.93 and 95%CI: 1.64–2.27) [25]. Others paid attention to the interaction of reperfusion and collateral status, and a previous study indicated that the effect of reperfusion on clinical outcome could be different depending on collateral status [26]. However, other studies showed opposite results. After a mean follow-up period of 5.2 months, no significant association was found between collateral status (OR: 1.681 and 95% CI: 0.683–4.140) and successful reperfusion in an observational study [19]. The data of our study supported that, in patients with ischemic stroke after mechanical thrombectomy, the pretreatment collateral status was associated with successful reperfusion and improved clinical outcomes.

A convincing hypothesis is that good collateral status sustains ischemic penumbra until reperfusion occurs, preventing the growth of cerebral infarction [16]. In accordance with the above finding, growth of cerebral infarction was found in individuals with poor collateral status [27]. In addition, patients with poor collateral status had almost 3 times higher rates of symptomatic intracerebral hemorrhage (sICH) compared to those with good collateral status [28].

Other factors were reported to affect the association of collateral status and clinical outcomes. In the data of the SOLITAIRE FR with the intention for thrombectomy (SWIFT) trial, the status of collateral circulation was strongly affected by the time from stroke onset to hospital arrival, with a mean time of 54 ± 16 min in grade 4 of collateral status and 232 ± 84 min in grade 0–1 [29]. Another study including 209 patients also showed the results that delayed collateral recruitment seemed to be different from early recruitment and may result in worse outcomes [30]. In our study, we found that there were interactions between previous ischemic stroke and statin use with collateral status on functional outcomes in subgroup analyses, whereas the effects of better collateral status on improved scores of mRS persisted in different ages, SBP and NIHSS at hospital arrival, and location of intracranial artery occlusion subgroups.

Animal studies have elucidated the major role of genetic variants in the number and diameter of collateral status and the degree of collateral remodeling. The extent of pial collateral in the brain varies over a 50-fold variation among different inbred mouse strains [31]. Dce1, a 737-Kb region, was identified to account for over 80% of the discrepancy in collateral status and the size of cerebral infarction after permanent ischemia among the C57BL/6 strain [32]. Besides, endothelial nitric oxide synthase has been implicated to play a role in forming native collateral and in collateral remodeling [33].

Due to the favorable clinical outcome in patients with better collateral status, attention has been paid to the adjunctive therapeutic augmentation of collateral circulation that might be beneficial for patients with ischemic stroke. A preclinical study found that mild hypertension induced by pharmacy could augment pial collateral flow, which led to improved blood flow and oxygen metabolism in the ischemic core and penumbra [34]. Besides, a study in mice indicated that statin, a cholesterol-lowering drug, upregulated the expression and activity of endothelial nitric oxide (NO) and augmented cerebral blood flow, preventing cerebral infarction and improving neurological function [35]. A subsequent clinical study supported that premorbid use of statins was significantly associated with excellent collateral status (OR: 7.841 and 95% CI: 1.96–31.363) [36]. The abovementioned association was consistent with the finding of our study, indicating that statin use may contribute to the effect of collateral status on good mRS.

The study has several limitations. First, due to a lack of standardization of collateral status as assessed by the CTA, we could not avoid subjective bias when the data of the CTA was judged by two neurologists. However, a third reader might help solve the difference between these two neurologists. Second, the interaction of history of ischemic stroke and statin use with collateral status must be interpreted with caution due to the small sample size. The third limitation is the observational design of our study; thus, randomized clinical trials are needed to demonstrate the causal relation between collateral status and clinical outcomes. However, as far as we know, there is no large clinical trial to verify the relationship. In the future, we believe that randomized clinical trials will demonstrate the causal relation of collateral status with mRS and death.

In conclusion, among patients with acute ischemic stroke caused by the anterior circulation occlusion, good collateral status is associated with greater reperfusion, higher scores on mRS, and lower mortality after mechanical thrombectomy.

## Figures and Tables

**Figure 1:** Degree of reperfusion stratified by collateral status (0, 1, 2, 3). The mTICI 0/1/2a was defined as unsuccessful reperfusion, and the mTICI 2b/3 as successful reperfusion.

**Figure 2:** Distribution of functional outcomes at 90 days (poor collaterals versus good collaterals). Functional outcomes were estimated by the scores on the modified Rankin scale ranging from 0 to 6.

**Table 1:** Characteristics of patients by collateral status.

Variables	Poor collaterals (*n* = 109)	Good collaterals (*n* = 110)	*P* value
Age, mean ± SD (yrs)	68.1 ± 10.7	67.2 ± 7.4	0.240
Male, *n* (%)	57 (52.3)	61 (55.5)	0.171
History of diseases, *n* (%)			
Hypertension	79 (72.5)	72 (65.5)	0.025
Diabetes	37 (33.9)	27 (24.5)	0.001
Atrial fibrillation	39 (35.8)	32 (29.1)	0.076
Ischemic stroke	21 (19.3)	13 (11.8)	0.005
Medication use, *n* (%)			
Statin	63 (57.8)	75 (68.2)	0.001
Antiplatelet	57 (52.3)	65 (59.1)	0.112
Anticoagulant	27 (24.8)	20 (18.2)	0.075
SBP at hospital arrival, median (IQR) (mmHg)	150.9 (25.2)	144.0 (25.1)	<0.001
Glucose at hospital arrival, median (IQR) (mmol/L)	7.5 (5.0–10.2)	7.0 (5.4–8.7)	0.231
Time from stroke onset to intravenous alteplase, median (IQR) (min)	125 (82–167)	117 (74–152)	0.354
Time from stroke onset to groin puncture, median (IQR) (min)	245 (205–289)	258 (25–309)	0.245
Time from stroke onset to revascularization, median (IQR) (min)	321 (271–376)	340 (277–387)	0.192
Location of intracranial artery occlusion, *n* (%)			<0.001
Intracranial ICA	39 (35.8)	34 (30.9)	
M1 segment	58 (53.2)	65 (59.1)	
M2 segment	12 (11.0)	11 (10.0)	
NIHSS at hospital arrival, median (IQR)	20 (16–24)	16 (13–20)	0.001
Good mRS (≤2) at 90 days, *n* (%)	52 (47.7)	64 (58.2)	<0.001
Mortality at 90 days, *n* (%)	29 (26.6)	22 (20.0)	0.003

**Table 2:** Association of collateral status and clinical outcomes.

Clinical outcomes	Poor collaterals (*n* = 109)	Good collaterals (*n* = 110)	Adjusted ORs (95%CI)	*P* value
mRS at 90 days, *n* (%)				
0–1	28 (25.7)	38 (34.5)	4.55 (3.17 to 7.24)	<0.001
0–2	52 (47.7)	64 (58.1)	4.28 (3.02 to 6.57)	<0.001
0–3	62 (56.9)	73 (66.3)	3.65 (2.15 to 6.03)	<0.001
0–4	72 (66.1)	81 (73.6)	2.10 (1.25 to 4.37)	0.001
Death at 90 days, *n* (%)	29 (26.6)	22 (20.0)	0.87 (0.72 to 0.96)	0.012

Odds ratios (ORs) were adjusted for age, history of diseases, medication use, SBP at hospital arrival, location of intracranial artery occlusion, and the NIHSS at hospital arrival.

**Table 3:** Subgroup analysis of the effect of collateral status on good mRS (≤2).

Subgroup	Number of patients	ORs (95%CI)	*P* value for interaction
Age (yrs)			0.192
<65 yr	81	4.69 (3.18 to 7.80)	
≥65 yr	138	3.95 (2.94 to 6.75)	
History of ischemic stroke			0.002
Yes	34	7.81 (2.34, 19.21)	
No	185	3.47 (2.88, 5.47)	
Statin use			0.021
Yes	138	4.77 (3.78, 7.01)	
No	81	3.42 (1.99, 7.51)	
SBP at hospital arrival			0.85
<140 mmHg	68	4.02 (1.94, 7.04)	
≥140 mmHg	151	3.98 (2.37, 6.96)	
NIHSS at hospital arrival			0.174
5–15	71	3.57 (1.78, 6.47)	
≥16	148	3.94 (2.14, 5.17)	
Location of intracranial artery occlusion			0.090
Intracranial ICA	73	3.94 (1.85, 7.02)	
M1 segment	123	4.01 (2.57, 6.11)	
M2 segment	23	9.51 (1.04, 19.17)	

## Data Availability

The analysed data sets generated during the study are available from the corresponding author on reasonable request.

## References

[1] Wang W., Jiang B., Sun H. (2017). Prevalence, incidence, and mortality of stroke in China. *Circulation*.

[2] Johnston S. C., Mendis S., Mathers C. D. (2009). Global variation in stroke burden and mortality: estimates from monitoring, surveillance, and modelling. *The Lancet Neurology*.

[3] Wang Z., Li J., Wang C. (2013). Gender differences in 1-year clinical characteristics and outcomes after stroke: results from the China National Stroke Registry. *PLoS One*.

[4] Cucchiara B., Elm J., Easton J. D. (2020). Disability after minor stroke and transient ischemic attack in the POINT trial. *Stroke*.

[5] Goyal M., Demchuk A. M., Menon B. K. (2015). Randomized assessment of rapid endovascular treatment of ischemic stroke. *New England Journal of Medicine*.

[6] Berkhemer O. A., Fransen P. S. S., Beumer D. (2015). A randomized trial of intraarterial treatment for acute ischemic stroke. *New England Journal of Medicine*.

[7] Saver J. L., Goyal M., Bonafe A. (2015). Stent-retriever thrombectomy after intravenous t-PA vs. t-PA alone in stroke. *New England Journal of Medicine*.

[8] Jovin T. G., Chamorro A., Cobo E. (2015). Thrombectomy within 8 hours after symptom onset in ischemic stroke. *New England Journal of Medicine*.

[9] Albers G. W., Marks M. P., Kemp S. (2018). Thrombectomy for stroke at 6 to 16 hours with selection by perfusion imaging. *New England Journal of Medicine*.

[10] Nogueira R. G., Jadhav A. P., Haussen D. C. (2018). Thrombectomy 6 to 24 hours after stroke with a mismatch between deficit and infarct. *New England Journal of Medicine*.

[11] Ginsberg M. D. (2018). The cerebral collateral circulation: relevance to pathophysiology and treatment of stroke. *Neuropharmacology*.

[12] Hartkamp M. J., van Der Grond J., van Everdingen K. J., Hillen B., Mali W. P. T. M. (1999). Circle of Willis collateral flow investigated by magnetic resonance angiography. *Stroke*.

[13] Sheth S. A., Sanossian N., Hao Q. (2016). Collateral flow as causative of good outcomes in endovascular stroke therapy. *Journal of Neurointerventional Surgery*.

[14] Kim B. J., Chung J.-W., Park H.-K. (2017). CT angiography of collateral vessels and outcomes in endovascular-treated acute ischemic stroke patients. *Journal of Clinical Neurology*.

[15] Park J.-S., Kwak H.-S., Chung G. H., Hwang S. (2018). The prognostic value of CT-angiographic parameters after reperfusion therapy in acute ischemic stroke patients with internal carotid artery terminus occlusion: leptomeningeal collateral status and clot burden score. *Journal of Stroke and Cerebrovascular Diseases*.

[16] Jung S., Gilgen M., Slotboom J. (2013). Factors that determine penumbral tissue loss in acute ischaemic stroke. *Brain*.

[17] Jansen I. G., Mulder M. J., Goldhoorn R.-J. B. (2019). Impact of single phase CT angiography collateral status on functional outcome over time: results from the MR CLEAN Registry. *Journal of Neurointerventional Surgery*.

[18] Liebeskind D. S., Jahan R., Nogueira R. G., Zaidat O. O., Saver J. L. (2014). Impact of collaterals on successful revascularization in solitaire FR with the intention for thrombectomy. *Stroke*.

[19] Nordmeyer H., Webering N., Chapot R. (2017). The association between collateral status, recanalization and long term outcome in stroke patients treated with stent retrievers - are there indications not to perform thrombectomy based on CT angiography?. *Journal of Neuroradiology*.

[20] Powers W. J., Rabinstein A. A., Ackerson T. (2018). 2018 guidelines for the early management of patients with acute ischemic stroke: a guideline for healthcare professionals from the American Heart association/American stroke association. *Stroke*.

[21] Tan I. Y. L., Demchuk A. M., Hopyan J. (2009). CT angiography clot burden score and collateral score: correlation with clinical and radiologic outcomes in acute middle cerebral artery infarct. *American Journal of Neuroradiology*.

[22] Zaidat O. O., Yoo A. J., Khatri P. (2013). Recommendations on angiographic revascularization grading standards for acute ischemic stroke. *Stroke*.

[23] Saver J. L. (2007). Novel end point analytic techniques and interpreting shifts across the entire range of outcome scales in acute stroke trials. *Stroke*.

[24] Menon B. K., Qazi E., Nambiar V. (2015). Differential effect of baseline computed tomographic angiography collaterals on clinical outcome in patients enrolled in the interventional management of stroke III trial. *Stroke*.

[25] Qian J., Fan L., Zhang W., Wang J., Qiu J., Wang Y. (2020). A meta‐analysis of collateral status and outcomes of mechanical thrombectomy. *Acta Neurologica Scandinavica*.

[26] Nambiar V., Sohn S. I., Almekhlafi M. A. (2014). CTA collateral status and response to recanalization in patients with acute ischemic stroke. *American Journal of Neuroradiology*.

[27] Bang O. Y., Saver J. L., Kim S. J. (2011). Collateral flow predicts response to endovascular therapy for acute ischemic stroke. *Stroke*.

[28] Chuang Y.-M., Chan L., Lai Y.-J. (2013). Configuration of the circle of Willis is associated with less symptomatic intracerebral hemorrhage in ischemic stroke patients treated with intravenous thrombolysis. *Journal of Critical Care*.

[29] Liebeskind D. S., Jahan R., Nogueira R. G. (2016). Early arrival at the emergency department is associated with better collaterals, smaller established infarcts and better clinical outcomes with endovascular stroke therapy: SWIFT study. *Journal of Neurointerventional Surgery*.

[30] Yeo L. L. L., Paliwal P., Low A. F. (2016). How temporal evolution of intracranial collaterals in acute stroke affects clinical outcomes. *Neurology*.

[31] Wang S., Zhang H., Wiltshire T., Sealock R., Faber J. E. (2012). Genetic dissection of the Canq1 locus governing variation in extent of the collateral circulation. *PLoS One*.

[32] Sealock R., Zhang H., Lucitti J. L., Moore S. M., Faber J. E. (2014). Congenic fine-mapping identifies a major causal locus for variation in the native collateral circulation and ischemic injury in brain and lower extremity. *Circulation Research*.

[33] Dai X., Faber J. E. (2010). Endothelial nitric oxide synthase deficiency causes collateral vessel rarefaction and impairs activation of a cell cycle gene network during arteriogenesis. *Circulation Research*.

[34] Shin H. K., Nishimura M., Jones P. B. (2008). Mild induced hypertension improves blood flow and oxygen metabolism in transient focal cerebral ischemia. *Stroke*.

[35] Laufs U., Gertz K., Dirnagl U., Böhm M., Nickenig G., Endres M. (2002). Rosuvastatin, a new HMG-CoA reductase inhibitor, upregulates endothelial nitric oxide synthase and protects from ischemic stroke in mice. *Brain Research*.

[36] Lee M. J., Bang O. Y., Kim S. J. (2014). Role of statin in atrial fibrillation-related stroke: an angiographic study for collateral flow. *Cerebrovascular Diseases*.

